# Potential Use of Anti-Cancer Drugs for Treatment of Preeclampsia by Targeting the miRNA-IGF1R-PI3K-AKT Axis

This article has been retracted.

**DOI:** 10.1155/2022/3883082

**Published:** 2022-08-22

**Authors:** Jieyan Li, Lei Hou, Rong Zhao, Liying Zou

**Affiliations:** Department of Obstetrics, Beijing Obstetrics and Gynecology Hospital, Capital Medical University, Beijing Maternal and Child Health Care Hospital, No. 251 Yaojiayuan Road Chaoyang, Beijing 100026, China

## Abstract

**Aim:**

Preeclampsia (PE) belongs to hypertensive disorders of pregnancy (HDP), which can cause maternal death worldwide. This study aimed to identify the miRNA-mRNA-associated ceRNA network and to find new treatment schedules for PE.

**Methods:**

4 microarray datasets were downloaded from the Gene Expression Omnibus database. We obtained 1737 differentially expressed mRNAs (865 upregulated and 872 downregulated) and 148 differentially expressed miRNAs (76 upregulated and 72 downregulated) from the placenta tissues of PE, respectively. Functional enrichment analyses of DEmRNAs were performed. The regulatory relationship between DEmiRNAs and DEmRNA was predicted via related databases. An miRNA-mRNA regulatory network was constructed.

**Results:**

hsa-let-7c and IGF1R were identified as potential regulators for PE, and function enrichment analysis showed that the PI3K-Akt signaling pathway was closely related. Therefore, ceRNAs might regulate the PI3K-Akt signaling pathway via the upregulation of IGF1R by binding to hsa-let-7c, affecting invasion of trophoblast, angiogenesis, and proinflammation in PE. Further study demonstrated that anticancer drugs including the PI3K inhibitor, AKT inhibitor, and IGF-1 inhibitor might be a potential solution for PE treatment.

**Conclusions:**

The hsa-let-7c/IGF1R axis might affect the PI3K-Akt signaling pathway which is involved in the pathogenesis of PE, and inhibitors targeting this pathway might be used for PE treatment.

## 1. Introduction

Preeclampsia (PE) belongs to hypertensive disorders of pregnancy (HDP), affecting 5% to 7% of all pregnant women and is associated with more than 70000 maternal deaths and 500000 fetal deaths around the world every year [1]. According to the International Society for the Study of Hypertension in Pregnancy (ISSHP), PE is defined as the presence of new-onset hypertension (≥140/90 mmHg) after 20 weeks' gestation accompanied by proteinuria or evidence of maternal acute kidney injury, liver dysfunction, neurological features, hemolysis or thrombocytopenia, or fetal growth restriction (FGR) [2]. The precise etiology of PE remains controversial. However, the placenta is considered to be central to the pathogenesis by previous clinical and pathological studies. The pathogenesis of PE is generally recognized to have 2 stages: at the first stage, insufficient placental trophoblast cell invasion leads to placental hypoperfusion; at the second stage, poor placental perfusion leads to release of growth factors, cytokines, inflammatory factors, steroids hormones, neuropeptide hormones, etc., in the local microenvironmental and causing PE [1, 3–6]. Despite these extensive studies on PE, no more effective treatment than delivery has been developed [7]. The exact pathogenesis remains to be elucidated.

MicroRNAs (miRNAs) are short, noncoding RNA molecules, acting as key regulators of gene expression programs. The important roles of miRNAs have been demonstrated during many pathophysiological processes, such as immune cell development, angiogenesis, and cell proliferation and adhesion [8]. Several studies have revealed that miRNAs may regulate trophoblast cell invasion (miRNA-181a-5p, miRNA-155, miRNA-223, miRNA-148a, and miRNA-152) and migration (miRNA-210), angiogenesis (miRNA-144-3p, miRNA-155), and the inflammation-related pathway (miRNA-155, miRNA-210) in PE [9–12]. In addition, a single miRNA can regulate many target genes in PE. For example, miRNA-181a-5p was observed to be overexpressed in human preeclamptic placentas compared with healthy controls. And metalloproteinases 2, 9 (MMP2 and MMP9) and insulin-like growth factor 2 mRNA-binding protein 2 (IGF2BP2) were shown to be the target genes of miRNA-181a-5p [13, 14]. However, the conclusions derived from all these studies have been limited by sample size and heterogeneity.

In the present study, we aimed to identify the key genes and microRNAs in PE by reanalyzing multiple datasets from the Gene Expression Omnibus (GEO) database. We found that hsa-let-7c-5p was involved in PE by regulating IGF1R expression and its downstream PI3K/AKT pathway, which might modulate invasion of trophoblast, angiogenesis, and proinflammation. This finding may provide a new target for the diagnosis and treatment of PE.

## 2. Materials and Methods

### 2.1. Retrieval and Process of Data

The mRNAs and miRNAs expression levels of placental tissue samples from PE patients and healthy parturient women were downloaded from the GEO database, GSE114349, GSE177049, GSE148241, and GSE168860). The details are shown in Table 1. 

### 2.2. Differentially Expressed mRNA and miRNA Analysis

The software edgeR was used to screen the differentially expressed mRNAs (DEmRNAs). *P* value <0.05 and |log2FC| ≥1 were chosen as the cut-off thresholds. To screen differentially expressed miRNAs (DEmiRNAs) between PE and normal placental tissue, limma was successively conducted, with the *P* value < 0.05 and |log2FC|>0.5 as the cut-off criterion. Volcano plots for the visualization of differentially expressed genes were generated using the *R* package “EnhancedVolcano”. Heatmaps of the gene expression were plotted using the *R* package “heatmap”.

### 2.3. Functional Enrichment Analysis

Differentially expressed genes were selected as input to perform gene functional enrichment analysis through DAVID (https://david.ncifcrf.gov/) and Metascape (http://metascape.org/gp/index.html#/main/step1). Gene Ontology (GO) and Kyoto Encyclopedia of Genes and Genomes (KEGG) pathway analysis of upregulated and downregulated genes were performed. GO analysis included biological process (BP), cellular component (CC), and molecular function (MF) enrichment analyses were performed. The KEGG database is a knowledge base for systematic analysis, annotation, and visualization of gene functions.

### 2.4. Targeted Genes of the miRNAs and miRNA-mRNA Network

The potential miRNA targets were identified using miRDB (http://www.mirdb.org/) and miRWalk (http://129.206.7.150/) with default settings. The intersection set of the results of the two methods was used for further analyses. The complex integrated networks of miRNA–mRNAs were constructed by using Cytoscape (v3.7.1, https://cytoscape. org). The dataset GSE177049 was used to validate the results.

### 2.5. Drug Sensitivity Prediction

The online web-based tool (https://clue.io/) was used to analyze the potential treatment options for PE treatment. Briefly, both upregulated genes and downregulated gene lists were uploaded to the website, followed by interactive analysis of similar gene expression signatures upon treatment with compounds.

## 3. Results

### 3.1. Differential Expression Analysis

To investigate the gene expression pattern in preeclampsia patients, transcriptome data between placenta tissue of preeclampsia patients and healthy tissues were analyzed. As shown in Figures 1(a) and 1(c), 1737 DEmRNAs (865 upregulated and 872 downregulated) were identified in the GSE148241 dataset (Figure 1(a)) and 148 DEmiRNAs (76 upregulated and 72 downregulated) were identified in the GSE14349 dataset, respectively. In addition, the top 50 DEmRNAs (Figure 1(b)) and DEmiRNAs (Figure 1(d)) are exhibited in heatmaps.

### 3.2. Functional Enrichment Analysis

To better understand the major function of DEmRNAs in PE, we conducted GO enrichment and KEGG pathway analysis (Figure 2). We found that upregulated genes in PE were mainly enriched for hormone-related pathway, immune and phosphatidylinositol 3-kinase signaling, such as the estrogen signaling pathway, inflammatory response, response to hypoxia, metal ion transport, cellular response to cytokine stimulus, positive regulation of phosphatidylinositol 3-kinase activity, and signaling (Figures 2(a) and 2(b)). Whereas, genes downregulated in PE were enriched for pathways including oxygen transporter activity, PI3K-Akt signaling pathway, calcium signaling pathway, oxytocin signaling pathway, and so on (Figures 2(b) and 2(c)). Interestingly, some pathways, such as the PI3K signaling pathway and calcium signaling pathway were significantly enriched in both upregulated and downregulated genes, which might predict complex regulation.

To directly assess the role of miRNA dysregulation in PE, we next conducted the miRNA-mRNA interaction network. Upregulated DEmiRNAs (*n* = 56) and their targeted downregulated DEmRNAs (*n* = 152) are shown in Figure 3(a). Downregulated DEmiRNAs (*n* = 63) and their targeted upregulated DEmRNAs (*n* = 227) are shown in Figure 3(b). To determine the functions of the targeted genes of miRNAs, functional enrichment analysis was performed using DAVID. We found that VEGF signaling pathway, MAPK signaling pathway, HIF-1 signaling pathway, PI3K-Akt signaling pathway, and insulin signaling pathway were significantly enriched. To further determine the key miRNA and targeted genes, Venn diagrams showed the intersection between exploratory datasets (mRNA: GSE148241; miRNA: GSE114349) and GSE177049. The details can be found in Supplementary Table S1. hsa-let-7c-5p/IGFR1 and hsa-miR-193b-3p/ZMAT3 were consistent in both datasets (Figure 4). We have also explored the expression of hsa-let-7c in plasma, and found that hsa-let-7c expression in PE was lower than that in the control group, whereas the difference did not reach significance (Figure S1(a)). Another homolog such as hsa-let-7c-5p in PE was lower than that in the control group (Figure S1(b)). The difference was not significant. In the placenta tissue of PE, hsa-let-7a-5p, hsa-let-7b-5p, hsa-let-7e-5p, and hsa-let-7f-2-3p were significantly downregulated in GSE114349 (Figure S1(c)). In the GSE177049, hsa-let-7a-5p, hsa-let-7b-3p, hsa-let-7c-5p, hsa-let-7d-3p, hsa-let-7d-5p, hsa-let-7f-2-3p, hsa-let-7f-5p, hsa-let-7g-5p was downregulated in PE (Figure S1(d)).

### 3.3. In Silico Analysis Revealed Potential Drugs for PE Treatment

Accumulated transcriptome data upon treatment with various compounds has enabled the prediction of drug sensitivity according to the differentially expressed gene signatures. To this end, both upregulated genes and downregulated gene signatures were used to predict potential treatment options for PE patients. The results demonstrated that antagonists targeting the IGF1R-PI3K pathway might be candidates for PE treatment, which is consistent with the activation of this pathway in PE tissue as evidenced by the bioinformatic analysis. Besides, inhibitors for EGFR and MAPK might be also listed as candidates for PE treatment (Table 2).

## 4. Discussion

PE is a common and serious gestational hypertension, characterized by complexity and multifactorial pathogenesis [15]. Because of its possible condition such as eclampsia, HELLP syndrome, placental abruption [16], early detection, and timely intervention, adequate and proper prenatal care is critical for PE. However, at the first stage of PE, clinical symptoms are usually not obvious. When the disease comes to the second stage, adverse effects to the mother and child have already happened. Therefore, new targets for the prediction and earlier diagnosis and treatment of PE need to be researched.

The functional pattern of the miRNA–mRNA regulatory network has been shown in the pathomechanisms of PE. Moreover, a lot of studies about miRNA and mRNA expression profiles in PE were published [17–19]. However, small sample sizes, different sample origins, and data processing may cause inconsistent results. In this present work, we identified a potential miRNA–mRNA regulatory pathway in PE. By integrative analysis of multiple datasets, we identified that downregulated let-7c-5p and upregulated IGF1R were relatively stable. Our finding confirms similar results from previous studies. Angelika V. Timofeev demonstrated that a more than two-fold decrease in let-7c-5p expression levels was observed in the placenta of PE [20]. The expression of IGF1R was found to be downregulated in the preeclampsia placentas compared with controls [21]. In addition, we identified IGF1R as a let-7c-5p target gene by using the miRDB and miRWalk database. hsa-let-7c can bind to the IGF-1R 3′-UTR and inhibit the expression of IGF-1R mRNA, thereby suppressing IGF-1-induced signaling pathways and biological processes [22, 23].

hsa-let-7c is one member of the let-7 family, which maps to human chromosome 21q11-21. hsa-let-7 miRNA plays an important role in regulating cell proliferation and differentiation, especially in cancers [24]. The let-7 family is among the earliest microRNAs found. Recent studies have indicated that it is highly expressed in many systems, including cerebral and cardiovascular systems. Numerous researches have implicated the aberrant expression of let-7 members in cardiovascular diseases, such as stroke, cardiac fibrosis, and atherosclerosis, as well as in inflammation related to these diseases [25]. However, the role of hsa-let-7c/IGF1R in PE was rarely reported. Thus, we performed functional enrichment analyses to detect the potential signaling pathway in PE. We found that the PI3K/Akt signaling pathway and MAPK pathway were enriched not only in DEmRNAs but also in DEmiRNA-target genes. IGF1R is a transmembrane tyrosine kinase-containing receptor. In general, IGF1 mediates cell behaviors via the IGF1R. Following binding of the IGF-1 ligand, IGF1R can activate downstream signaling pathways. Interestingly, PI3K/Akt and MAPK pathways are the major pathways downstream of the IGF/IGF1R axis [22]. It is therefore likely that such connections exist between hsa-let-7c and IGF1R/PI3K/Akt. The PI3K/Akt signaling pathways are common to PE and play key roles in many cellular processes [26], such as invasion of trophoblast [27], angiogenesis [28], and pro-inflammation [29]. Park JK demonstrated that inhibition of the PI3K-Akt pathway may decrease sFlt1 secretion in human placental hypoxia models, which provides a useful therapeutic approach for PE [30].

There are many drugs currently being assessed to treat PE, including proton pump inhibitors (PPIs), metformin, melatonin, statins, sofalcone, resveratrol, sulfasalazine, and sildenafil citrate. These drugs show positive effects in preclinical studies, targeting placental and endothelial dysfunction. However, novel therapeutics can raise safety concerns for the developing fetus. Combining targeted drug delivery with effective therapeutics could be the future of preeclampsia treatment [31]. Our data also supported the proposed treatment of PE patients with PI3K-AKT pathway inhibitors. Furthermore, single or combined use of antagonists for blocking the upstream or downstream factors might be also considered as potential treatment options. Numerous Akt and IGF1R inhibitors have anticancer effects in preclinical investigation. However, the advances in clinical evaluation are somewhat slow. Many inhibitors have limited anti-cancer activity as a monotherapy in the clinic. And some drugs have some side effects including diarrhea, hypertension, rash, hyperglycemia and fatigue [32]. What is critically needed is the development of predictive biomarkers that can guide future research in applying this therapeutic strategy to the patient populations that is most likely to benefit [33]. In the present study, we explored a new signaling pathway between PI3K/Akt and PE. hsa-let-7c/IGF1R/PI3K/Akt might play an important role in the pathogenesis of PE. However, such a hypothesis requires further validation by experimental investigations.

## 5. Conclusions

By comprehensive bioinformatics analysis, we found that hsa-let-7c and IGF1R were the key genes in the miRNA-mRNA networks of PE. The hsa-let-7c/IGF1R axis might affect the PI3K-Akt signaling pathway which is involved in the pathogenesis of PE, including invasion of trophoblast, angiogenesis, and proinflammation. This discovery might provide some new light on the mechanism of PE progression.

## Figures and Tables

**Figure 1:** The expressions of differentially expressed mRNAs and miRNAs. Volcano plots of (a) mRNA from GSE148241 and (c) miRNA from GSE114349. Heatmaps of (b) mRNA from GSE148241 and (d) miRNA from GSE114349. Red and blue indicate upregulation and downregulation, respectively.

**Figure 2:** Functional enrichment analysis. (a) GO term and KEGG pathway analyses of upregulated DEmRNAs by DAVID. (b) GO term and KEGG pathway analyses of upregulated DEmRNAs by Metascape. (c) GO term and KEGG pathway analyses of downregulated DEmRNAs by DAVID. (d) GO term and KEGG pathway analyses of downregulated DEmRNAs by Metascape.

**Figure 3:** The miRNA-mRNA interaction network. (a) The interaction network of upregulated miRNA and downregulated mRNA. (b) The interaction network of downregulated miRNA and upregulated mRNA. (c) GO term and KEGG pathway analyses of DEmiRNA-target genes. (d) Venn diagram of the DEmiRNA-target genes of GSE148241 and GSE177049.

**Figure 4:** hsa-let-7c-5p might regulate IGF1R involved in the PI3K/AKT pathway. RNA-seq and microarray data showing the mRNA expression level of has-let-7c-5p and IGF1R in PE and normal placental tissue from the GEO database. (a) Levels of hsa-let-7c-5p expression in PE (*n* = 20) and control (*n* = 21) placental tissues (GSE114349) (*P*=0.008484054). (b) IGF1R mRNA levels in placental tissues of PE (*n* = 9) and normal (*n* = 34) from GSE148241 (*P* = 0.009579). (c) Levels of hsa-let-7c-5p expression in PE (*n* = 5) and control (*n* = 5) placental tissues (GSE177049) (*P*=0.009990581). (d) IGF1R mRNA levels in placental tissues of PE (*n* = 5) and normal (*n* = 5) from GSE177049 (*P*=0.021232). (e) Biological function of the miRNA-IGF1R-PI3K-AKT axis.

**Table 1:** The detailed information of the datasets.

Database	Source	Sample		Type	Platform
		Control	*P*E		
GSE114349	https://www.ncbi.nlm.nih.gov/geo/Query/acc.cgi?acc=GSE114349	21	40	Noncoding RNA	Illumina HiSeq 2000 (Homo sapiens)

GSE177049	https://www.ncbi.nlm.nih.gov/geo/Query/acc.cgi?acc=GSE177049	5	5	mRNA	Illumina NextSeq 500 (Homo sapiens)
		5	5	miRNA	Illumina NovaSeq 6000 (Homo sapiens)

GSE148241	https://www.ncbi.nlm.nih.gov/geo/Query/acc.cgi?acc=GSE148241	32	9	mRNA	Illumina HiSeq 2500 (Homo sapiens)

GSE168860	https://www.ncbi.nlm.nih.gov/geo/Query/acc.cgi?acc=GSE168860	4	5	miRNA	Qiagen Homo sapiens miScript II RT kit

**Table 2:** Plot of nanoparticle size with respect to time, recorded over a 90 s period. The error bars represent the standard deviation of measurements for 20 particles in five separate sample runs (*n* = 100).

Pert_iname	Cell_iname	Pert_idose	Pert_itime (h)	Moa	Target_name	TAG
AS-605240	LNCAP	1.11* μ*M	24	PI3K inhibitor	PIK3CG	−1.6199
GDC-0941	HME1	0.12* μ*M	3	PI3K inhibitor	PIK3CG|PIK3CA|PIK3CB|PIK3CD	−1.6038
Taselisib	BJAB	0.01* μ*M	24	PI3K inhibitor	PIK3CA|PIK3CB|PIK3CD|PIK3CG	−1.5581
Alpelisib	OCILY3	0.01* μ*M	24	PI3K inhibitor	PIK3CA|PIK3CB|PIK3CD|PIK3CG	−1.5362
SAR-245409	MDAMB231	0.04* μ*M	24	PI3K inhibitor	MTOR|PIK3CG	−1.5214
Buparlisib	MCF7	0.03* μ*M	24	PI3K inhibitor	PIK3CA|PIK3CG	−1.5214
XL-147	A549	0.125* μ*M	24	PI3K inhibitor	PIK3CG|PIK3CA|PIK3CD	−1.5164
Taselisib	OCILY19	0.01* μ*M	24	PI3K inhibitor	PIK3CA|PIK3CB|PIK3CD|PIK3CG	−1.5109
Idelalisib	HBL1	2.5* μ*M	24	PI3K inhibitor	PIK3CD|PIK3CG|CCL3|CCL4|PIK3CA|PIK3CB	−1.5063
AZD-5363	HA1E	2.22* μ*M	24	AKT inhibitor	AKT1|AKT2|AKT3	−1.5825
MK-2206	OCILY19	0.04* μ*M	4	AKT inhibitor	AKT1|AKT2|AKT3	−1.5567
GDC-0068	THP1	0.03* μ*M	24	AKT inhibitor	AKT1|AKT2|AKT3|CYP3A5|PRKG1	−1.5259
GDC-0068	A375	2.22* μ*M	24	AKT inhibitor	AKT1|AKT2|AKT3|CYP3A5|PRKG1	−1.5081
MK-2206	MCF10 A	0.12* μ*M	24	AKT inhibitor	AKT1|AKT2|AKT3	−1.5067
AZD-5363	PC3	1.11* μ*M	24	AKT inhibitor	AKT1|AKT2|AKT3	−1.502
TAK-285	HELA	0.08* μ*M	24	EGFR inhibitor	ERBB2|EGFR	−1.5618
Afatinib	AGS	1.11* μ*M	24	EGFR inhibitor	EGFR|ERBB2|ERBB4	−1.5531
AZD-9291	A375	1.11* μ*M	24	EGFR inhibitor	EGFR	−1.5492
Erlotinib	MCF10 A	3.33* μ*M	24	EGFR inhibitor	EGFR|NR1I2	−1.5471
Erlotinib	MCF7	0.125* μ*M	24	EGFR inhibitor	EGFR|NR1I2	−1.5197
Gefitinib	K562	2.5* μ*M	24	EGFR inhibitor	EGFR|CYP2C19	−1.5159
Gefitinib	MCF7	0.37* μ*M	6	EGFR inhibitor	EGFR|CYP2C19	−1.5051
LY-2228820	A375	3.33* μ*M	24	P38 MAPK inhibitor	MAPK14	−1.6021
TAK-715	NPC	0.04* μ*M	24	P38 MAPK inhibitor	MAPK14|TNF	−1.6019
TAK-715	SKBR3	10* μ*M	24	P38 MAPK inhibitor	MAPK14|TNF	−1.5371
LY-2228820	HELA	0.08* μ*M	24	P38 MAPK inhibitor	MAPK14	−1.5273
TAK-715	MCF7	1.11* μ*M	6	P38 MAPK inhibitor	MAPK14|TNF	−1.5041

## Data Availability

https://www.ncbi.nlm.nih.gov/geo/query/acc.cgi?acc=GSE114349 https://www.ncbi.nlm.nih.gov/geo/query/acc.cgi?acc= GSE177049 https://www.ncbi.nlm.nih.gov/geo/query/acc.cgi?acc= GSE148241 https://www.ncbi.nlm.nih.gov/geo/query/acc.cgi?acc= GSE168860.

## Supplementary Materials

Supplementary Materials Figure S1. (a) Levels of hsa-let-7c-5p expression in PE (*n* = 5) and control (*n* = 4) plasma (GSE168860). (b) Levels of hsa-let-7a-5p expression in PE (*n* = 5) and control (*n* = 4) plasma (GSE168860). (c) Volcano plots of miRNA from GSE114349. (d) Volcano plots of miRNA from GSE177049. Table S1. The details of the Venn diagram in Figure 3(d) and 3(e).
